This article has been retracted.

# Effects of Periodontal Treatment on Levels of Proinflammatory Cytokines in Patients with Chronic Periodontitis: A Meta-Analysis

**DOI:** 10.1155/2022/9349598

**Published:** 2022-07-26

**Authors:** Jiahui Ren, Hong Li

**Affiliations:** Dental Department, Xi'an Union Hospital, Xi'an City, Shaanxi Province 710199, China

## Abstract

**Background:**

During the progression of chronic periodontitis (CP), changes in the levels of inflammatory factors are detected in serum and gingival sulcus fluid (GCF). The aim of this meta-analysis was to systematically evaluate the effect of periodontal treatment on GCF and serum proinflammatory cytokines (IL-6, TNF-*α*, and IL-8) in patients with CP.

**Methods:**

Literature searches were performed through PubMed, Web of Science, Embase, China National Knowledge Infrastructure (CNKI), and Wanfang Database. Randomized controlled trials comparing cytokine levels in periodontal treatment (experimental group) and control group between 2015 and 2020 were included.

**Results:**

There were a total of 13 studies included with 1220 patients. There were 630 cases in the experimental group and 590 cases in the control group. The meta-analysis showed that IL-6 levels in the GCF (SMD = −2.88, 95% CI (-3.68, -2.09), *P* < 0.001) and serum (SMD = −1.27, 95% CI (-1.72, -0.81), *P* < 0.001) were significantly lower in the experimental group compared with those before treatment. In addition, IL-8 levels in the GCF (SMD = −2.08, 95% CI (-3.40, -0.76), *P* < 0.001) and serum (SMD = −1.73, 95% CI (-2.76, -0.70), *P* < 0.001) were decreased after periodontal treatment, but more than that, a decrease was observed in TNF-*α* levels of GCF (SMD = −3.98, 95% CI (-5.23, -2.73), *P* < 0.001) and serum (SMD = −1.80, 95% CI (-3.16, -0.45), *P* < 0.001) after treatment.

**Conclusion:**

After periodontal therapy, the proinflammatory cytokines in the GCF and serum of patients with CP were significantly decreased compared with those before treatment, and the efficacy was remarkable.

## 1. Introduction

Periodontitis, as a common chronic inflammation that invades gingiva and periodontal tissues, is also an infectious disease characterized by progressive attachment loss and cementum loss [1]. In recent years, the incidence of chronic periodontitis (CP) has been up to 40% to 75% [2], and patients are getting younger. In particular, people in 35 to 44 years old have a 97.20% possibility of infecting CP [3]. Periodontitis not only leads to tooth loss but also increases the risk of atherosclerosis, adverse pregnancy outcomes, rheumatoid arthritis, aspiration pneumonia, and cancer [3].

Chronic inflammation is a complex biological process that occurs in response to infection or other triggers and leads to tissue damage [4]. Some subtypes of cytokines are proinflammatory mediators, also known as inflammatory cytokines such as interleukin (IL) and tumor necrosis factor (TNF). They play an important role in controlling inflammation and are closely related to periodontitis [5]. Studies have found that periodontitis damages present in two ways: direct destruction caused by periodontal pathogens or indirect destruction caused by host inflammatory response. The latter is the main pathway leading to periodontal tissue destruction [6, 7]. In the process of host response, a series of inflammatory mediators including IL and TNF play an important role. That is, they not only directly lead to the destruction of periodontal tissues but also affect the process of host inflammatory response to aggravate the destruction of periodontal tissues [8].

Studies have shown that basic periodontal therapy is currently the most effective treatment for CP, including instruction in oral hygiene, supragingival scaling, and subgingival scraping [9]. Several studies [10–12] have confirmed that periodontal treatment is able to effectively lower the levels of inflammatory factors such as IL-6, IL-8, and TNF-*α* in gingival crevicular fluid (GCF) and serum in patients with CP. However, due to the small sample size between studies, changes in inflammatory factor levels before and after treatment of CP cannot be accurately described. Therefore, in the current study, we systematically evaluated the changes of inflammatory cytokine levels in GCF and serum in patients with CP by including randomized controlled trials (RCT). In the meantime, we investigated the efficacy of periodontal treatment for CP.

## 2. Materials and Methods

### 2.1. Search Strategy

A systematic search based on scientific databases was conducted to obtain relevant theses, including PubMed, Web of Science, Embase, CNKI, and Wanfang Database. The search for medical subject heading terms and keywords was “periodontal treatment”, “chronic periodontitis”, “gingival crevicular fluid or GCF” or “serum”, and “cytokines”. Furthermore, an additional search of the reference lists from the relevant articles, conference papers, and abstracts was performed to dig out other potential articles.

### 2.2. Inclusion and Exclusion Criteria

We established the following criteria based on the PICOS model, namely, participants, interventions, comparison, outcomes, and study designs. (1) Participants (P): periodontal healthy patients diagnosed with CP according to medical diagnostic criteria and agreed to participate in the study in different departments of the same hospital and patients who were diagnosed as CP rather than aggressive periodontitis according to medical diagnostic criteria; patients must not receive periodontal therapy within at least half a year and take no hormones, antibiotics, and other drugs recently. (2) Interventions and comparisons (I, C): experimental group: patients receive basic periodontal treatment (oral hygiene instruction+supragingival plaque removal and subgingival scaling of tartar); control group: healthy individuals without periodontal disease who received body examination during the same period. Outcomes (O): levels of inflammatory factors IL-6, IL-8, and TNF-*α* in GCF as well as in serum. Study designs (S): all clinical studies were conducted to compare the differences in inflammatory factors in patients with CP treated with periodontal therapy and the control group.

Inclusion criteria were as follows: (1) patients in the experimental group met the diagnostic criteria for CP, while subjects in the control group should have no periodontal disease; (2) comparison was conducted between periodontal treatment and zero intervention; and (3) expound on the results of cytokines IL-6, IL-8, and TNF-*α* in the GCF or serum in patients.

Exclusion criteria were as follows: (1) the experimental group is not undergoing periodontal basic treatment or the control group is not treated without intervention; (2) review; (3) duplicate studies; and (4) data insufficiency, design flaws, and ambiguous conclusion. 13 literature were consequently included.

### 2.3. Quality Assessment and Data Extraction

The risk of bias in each identified study was assessed using the Cochrane Collaboration's tool [13]. The tool considered six different domains: (1) random sequence generation (selection bias); (2) allocation concealment (selection bias); (3) blinding of participants and personnel (performance bias); (4) blinding of outcome assessors (detection bias); (5) incomplete outcome data (attrition bias); and (6) selective reporting (reporting bias). Two researchers separately conducted quality assessment and data extraction. Meanwhile, they discussed and addressed issues about data extraction with the third researcher.

### 2.4. Statistical Analysis

Statistical analysis was performed using Stata16.0 software. Heterogeneity among studies was assessed using the Cochrane's *Q*-test and the *I*^2^ test. If the *Q*-test shows *P* < 0.05 or *I*^2^ test shows *I*^2^ > 50%, which indicates significant heterogeneity, the random effect model was conducted; otherwise, the fixed effect model was used. The results of numerical variable data were reported as standardized mean difference (SMD) with their 95% confidence interval (CI). *P* < 0.05 was considered statistically significant. Sensitivity analysis was conducted to evaluate the results of the meta-analysis.

## 3. Results

### 3.1. Baseline Characteristics of the Included Studies

Initially, there were a total of 736 articles being identified. Then, 61 articles were included after reviewing their titles, abstracts, and full texts. Finally, in view of study bias and research methods, 13 articles [10–12, 14–23] in Chinese met the selection criteria. These 13 eligible articles included 1220 patients, with 630 cases of periodontal therapy and 590 cases of the control group.  Table 1 shows the characteristics of the included studies, and Figure 1 shows the selection process of the eligible articles.

### 3.2. Result Analysis

#### 3.2.1. Changes of IL-6, TNF-*α*, and IL-8 in GCF

The outcome variable of 10 eligible articles [10–12, 14–16, 18, 20–22] displayed the IL-6 level in GCF. After data combination, it showed that the heterogeneity of the two indicators of each study was significant (*I*^2^ = 95.3%, *P* < 0.001). Therefore, the random effect model was performed. The meta-analysis showed that the IL-6 level of the experimental group in GCF was decreased after treatment, and the results (Figure 2(a)) had statistical differences (SMD = −2.88, 95% CI (-3.68, -2.09), *P* < 0.001).

Five trials [15, 18, 20, 22, 23] reported the IL-8 level in GCF from the experimental group, and the results demonstrated high heterogeneity (*I*^2^ = 97.0%, *P* < 0.001). A random effect model, therefore, was utilized for analysis. According to the meta-analysis, the experimental group of the TNF-*α* level in GCF was lower than that before treatment, and the results (Figure 2(b)) had statistical differences (SMD = −2.08, 95% CI (-3.40, -0.76), *P* < 0.001).

Nine included studies [10–12, 14, 15, 20–23] mentioned the TNF-*α* level in the GCF of the experimental group after treatment, and a high heterogeneity was shown (*I*^2^ = 97.7%, *P* < 0.001). Consequently, a random effect model was conducted which (Figure 2(c)) showed that the IL-8 level in GCF decreased significantly after treatment (SMD = −3.98, 95% CI (-5.23, -2.73), *P* < 0.001).

#### 3.2.2. Changes of IL-6, TNF-*α*, and IL-8 in Serum

The outcome variable in six studies [11, 15, 17–20] showed IL-6 levels in serum. With a combination of data, a significant heterogeneity was apparent (*I*^2^ = 83.9%, *P* < 0.001). Thus, a random effect model was used. The results of the meta-analysis showed that periodontal therapy could significantly reduce the serum IL-6 level in patients with CP, and the results (Figure 3(a)) were statistically significant (SMD = −1.27, 95% CI (-1.72, -0.81), *P* < 0.001).

There were three studies [15, 18, 20] investigating the serum IL-8 level after treatment in the experimental group, and the results had great heterogeneity (*I*^2^ = 92.0%, *P* < 0.001). The random effect model was consequently used for analysis. It was found (Figure 3(b)) that the serum TNF-*α* level after treatment in the experimental group was lower than that before treatment (SMD = −1.73, 95% CI (-2.76, -0.70), *P* < 0.001).

Five studies [11, 15, 17, 19, 20] evaluated the serum TNF-*α* level of an experimental group after treatment, and a significant heterogeneity could be seen (*I*^2^ = 97.5%, *P* < 0.001). Therefore, the random effect model was performed. The serum IL-8 level (Figure 3(c)) decreased significantly after treatment, according to the meta-analysis (SMD = −1.80, 95% CI (-3.16, -0.45), *P* < 0.001).

### 3.3. Sensitivity Analysis

The results of sensitivity analysis (Figures 4 and 5) indicated that the overall pooled results were not affected by excluding a single study even though altering the inclusion criteria, excluding low-quality studies, and removing the maximum weight and the minimum weight. Therefore, it could demonstrate that the results of this meta-analysis were credible with low sensitivity.

### 3.4. Publication Bias

It cannot confirm whether there is publication bias or not since each group of literature is less than ten. Thus, no funnel plot analysis is available.

## 4. Discussion

CP is a continuous inflammatory that alternates between a remission phase and an acute attack of inflammation [24]. The occurrence of CP is closely related to a variety of microorganisms in the oral cavity. Specifically speaking, microorganisms and their secretions such as lipopolysaccharide can enter the body through the damaged mucosal epithelium to activate humoral immunity and cellular immunity. Furthermore, microorganisms can stimulate mononuclear phagocyte to release inflammatory factors, which results in an increase in inflammatory cytokines such as IL-6, TNF-*α*, IL-5, and IL-8 [25, 26]. A total of 13 studies were included with similar study methods and high comparability. All studies showed that the levels of IL-6, IL-8, and TNF-*α* in the GCF as well as in the serum of the experimental group before treatment were higher than those of the control group, which was in accordance with the above study.

GCF is one kind of fluid that penetrates from the gingival connective tissue into the gingival sulcus, and its main component and function are similar to serum. Therefore, the changes in volume and content in GCF can be used to diagnose and treat periodontal diseases. Moreover, it is of great clinical significance to evaluate the curative effect.

According to the meta-analysis, the levels of IL-6, IL-8, and TNF-*α* in GCF and serum of the experimental group were significantly decreased after treatment. The results showed that after removing some periodontal stimulating factors through periodontal therapy, gingival inflammation was ameliorated, and the levels of IL-6, IL-8, and TNF-*α* inflammatory factors were reduced in GCF and serum, with statistically significant differences compared with the control group.

There were ten studies evaluating the difference of IL-6 level in GCF after periodontal therapy and six studies evaluating the difference of IL-6 level in serum after periodontal therapy. The meta-analysis showed that IL-6 in GCF as well as serum was significantly reduced after treatment. It has been reported that IL-6, a multifunctional proinflammatory cytokine, is synthesized against infection with a wide range of biological activities. IL-6 is closely related to antibody production, T-cell activation, B-cell differentiation, and osteoclast activation [27]. What is more, IL-6 leads to osteoclast differentiation and bone resorption, which are typical symptoms of CP [28]. As a potent inducer, it is revealed that IL-6 plays a role in catabolic effects on bone by mediating through osteoblasts/stromal cells, more specifically, through the regulation of RANKL and OPG expression in these cells [29]. Beyond that, the intensity of IL-6 expression is positively correlated with attachment loss [30], and IL-6 in CP is correlated with sustained tissue destruction [31]. Several studies have validated the association between IL-6 and the risk of periodontitis, which is in line with the meta-analysis in the current study. These results suggest that during the process of periodontal treatment, the level of IL-6 can be reduced so as to improve the gingival inflammatory. By ameliorating further periodontal damage caused by the inflammatory response, it is conducive to the treatment and recovery of CP.

Nine trials and five trials, respectively, reporting TNF-*α* levels in GCF as well as serum were included. The results pointed out that TNF-*α* levels in GCF as well as serum were lower after treatment. TNF-*α* is the most important endogenous induced proinflammatory factor in the inflammatory microenvironment of periodontal tissues. In the inflammatory microenvironment, TNF-*α* disrupts the homeostasis of bone remodeling, causes disturbance of bone metabolism, and accelerates the loss of bone tissue. Relevant studies [32] have confirmed that TNF-*α* can enhance bone fragmentation, inhibit osteogenesis, and destroy bone microarchitecture, which ultimately causes severe bone resorption and destruction. TNF-*α* can regulate osteogenic differentiation of BMSCs through a variety of pathways. Although there are various studies investigating this topic, researchers find it difficult to draw a consistent conclusion. They believe that TNF-*α* directly or indirectly regulates osteogenic differentiation of BMSCs through various signaling pathways such as Wnt signaling pathway, bone morphogenetic protein (BMP) signaling pathway, and MAPK signaling pathway. The meta-analysis in this study showed that the TNF-*α* levels in GCF and serum were significantly reduced after periodontal therapy. It indicates that in the time of receiving periodontal therapy, the level of TNF-*α* can be reduced. Therefore, the inflammatory response can be improved; the effect on bone tissue and damage can be reduced; and further periodontal damage can be avoided.

Five trials and three trials, respectively, reporting IL-8 levels in GCF as well as serum were eligible. The results revealed that there was a significant decrease in IL-8 levels in GCF as well as serum after treatment. Previous reports have confirmed that IL-8 levels play an important role in the etiology of CP. IL-8 factor is the most effective chemokine which is responsible for inducing cell chemotaxis, that is, directional migration of cells to inflammatory sites [33]. Chemokines are important for both the regulation of the inflammatory response and the ability to recruit and activate acute inflammatory cells. IL-8 factor also mediates the activation and migration of neutrophils which are the first line to resist periodontopathic bacteria that migrate from the peripheral blood into tissues [34]. After treatment, MMP-8 levels in salivary and GCF were significantly lower. Meanwhile, periodontal therapy can also reduce IL-8 levels as well as the inflammatory response.

Nevertheless, there are some limitations existing in this meta-analysis. First of all, with insufficient samples and study subjects, there may be some selection bias. Thus, the conclusion might not be universal among the overall population. Afterwards, the retrieval efficiency is low since there is only Chinese and English literature and the final articles included in the meta-analysis were all in Chinese. Furthermore, the study does not use allocation concealment scheme and blind method to control the information bias. Finally, there are many treatment methods for CP used in clinical practice. However, the experimental group in this study selected merely one basic periodontal therapy, which was not compared with other clinical protocols, such as antibacterial photodynamic therapy and semiconductor laser method. Besides, the treatment period is not strictly specified in this study, affecting the extrapolation of the results into clinical application.

## 5. Conclusion

In summary, the current results show that periodontal treatment is effective for patients with CP for it is conducive to improve the levels of IL-6, IL-8, and TNF-*α* cytokines in GCF and serum in patients with CP. With such excellent clinical efficacy, it is worthwhile to promote periodontal treatment.

## Figures and Tables

**Figure 1:** Flow diagram to show selection process.

**Figure 2:** Forest plots comparing the IL-6, IL-8, and TNF-*α* levels in the gingival crevicular fluid after treatment. (a) Interleukin- (IL-) 6 levels. (b) IL-8 levels. (c) Tumor necrosis factor- (TNF-) *α* levels.

**Figure 3:** Forest plots of serum IL-6 (a), IL-8 (b), and TNF-*α* (c) levels after treatment.

**Figure 4:** Meta-based sensitivity analysis for comparisons of IL-6 (a), IL-8 (b), and TNF-*α* (c) in the gingival crevicular fluid after periodontal treatment.

**Figure 5:** Meta-based sensitivity analysis for comparisons of IL-6 (a), IL-8 (b), and TNF-*α* (c) in serum after periodontal treatment.

**Table 1:** Baseline characteristics of the included studies.

No.	First author	Year	Sample time (year.month)	Diagnostic method	No. of patients treat/con	Age (years)	Sex ratio (male/female)	Study design	Outcome measured	
									Gingival crevicular fluid	Serum
1	Yu Qin	2018	2015.6~2017.10	ELISA	40/25	37.5 ± 5.6	23/17	Retrospective	IL-6; TNF-*α*	NR
2	Jia Ning	2020	2018.1~2018.12	ELISA	64/64	55.12 ± 2.39	39/25	Retrospective	IL-6; TNF-*α*	IL-6; TNF-*α*
3	Yuan Dan	2016	2014.1~2015.3	ELISA	43/43	56.9 ± 5.5	26/17	Retrospective	IL-6; TNF-*α*	NR
4	Chang Chunrong	2013	2007.7~2008.10	ELISA	40/50	NR	NR	Retrospective	IL-6; TNF-*α*	NR
5	Zhang Junqi	2018	2015.1~2017.12	ELISA	50/50	58.37 ± 5.16	32/18	Retrospective	IL-6; IL-8; TNF-*α*	IL-6; IL-8; TNF-*α*
6	Li Ming	2014	2011.1~2013.2	ELISA	40/40	34.50 ± 11.82	18/22	Retrospective	IL-6	NR
7	Wu Liuzhong	2014	2012.2~2013.9	ELISA	72/72	23~67	38/34	Retrospective	IL-6; TNF-*α*	NR
8	Liu Haitao	2018	2015.8~2016.12	ELISA	36/36	39.87 ± 10.21	19/17	Retrospective	IL-6; IL-8	IL-6; IL-8
9	Yu Jiangbo	2013	2012.1~2012.6	ELISA	32/0	45~65	15/17	Retrospective	IL-6; TNF-*α*	NR
10	Huang Haixia	2018	2015.9~2017.9	ELISA	46/43	48.6 ± 4.7	24/19	Retrospective	IL-6; IL-8; TNF-*α*	IL-6; IL-8; TNF-*α*
11	Wu Di	2017	2013.10~2015.11	ELISA	67/67	42.03 ± 6.94	37/30	Retrospective	NR	IL-6; TNF-*α*
12	Niu Jiahui	2018	2016.8~2017.7	ELISA	60/60	41.6 ± 7.8	33/27	Retrospective	NR	IL-6; IL-8; TNF-*α*
13	Li Feng	2018	2016.1~2017.1	ELISA	40/40	61.04 ± 2.15	25/15	Retrospective	NR	IL-8; TNF-*α*

Note: NR: not reported; Treat: treatment; Con: control.

## Data Availability

The data used to support the findings of this study are available from the corresponding author upon request.
